# Construction and Signal Feature Processing of Gold Nanobiosensors Based on the Internet of Things

**DOI:** 10.1155/2022/1432266

**Published:** 2022-01-10

**Authors:** Ling Chen

**Affiliations:** School of Life Sciences, Jiangsu University, Zhenjiang, Jiangsu 212013, China

## Abstract

With the continuous development of signal amplification technology and nanotechnology, more and more electrochemical sensors combining nanotechnology and signal amplification technology are applied in the field of analysis. In this paper, combined with the Internet of Things technology, the construction of gold nanobiosensors and signal characteristic processing are carried out. In this paper, a T-rich DNA probe is used as the recognition element, modified on the electrode surface, combined with DNA-modified nanogold particle amplification technology, and the electroactive substance peg amine is used as the signal molecule to develop a highly sensitive electrochemical biosensor for the detection of melamine. The sensor has good specificity and sensitivity, and the detection limit is as low as 0.5 NM. In addition, by combining sensors with the Internet of Things technology, melamine monitoring and signal characteristic processing can be carried out in real time. This model can easily achieve the purpose of accurate and quantitative analysis of melamine toxins and can be effective for food safety.

## 1. Introduction

Traditional sensing technology has some shortcomings in sensitivity, response time, equipment maintenance, etc. Therefore, the development of a simpler, faster, and more sensitive sensor has always been one of the research hotspots [1, 2]. Nanogold has unique properties such as strong surface effect, good biocompatibility, and excellent heat conduction effect. Compared with other nanomaterials, it is easy to prepare. Therefore, sensors based on nanogold can be widely used in biology, environment, medicine, and other fields [1, 3]. The research and application of the combination of nanomaterials and biosensors involves many disciplines such as biotechnology, information technology, and rice sciences. At the same time, the research of nanomaterials in biosensors provides many innovative research ideas for basic research. It has attracted more and more attention from all walks of life in the world and has become the frontier and hot spot of scientific research [4, 5]. Therefore, at the same time, the development and application of the combination of the two also has an important impact on clinical testing, medical diagnosis, environmental monitoring, and other fields and has also obtained unprecedented development opportunities [6].

Electrochemical biosensors are established on the basis of biosensors, using biological materials as sensitive parts, and various electrode materials as converters, which are converted into electrochemical signals to achieve detection purposes [7–9]. Electrochemical biosensors have broad application prospects in biomedicine, environmental monitoring, food industry, and other fields due to their high sensitivity, good selectivity, and rapidity [10]. Some scholars have developed a new type of electrochemical sensor to realize the detection of DNA based on the cyclic amplification of target DNA assisted by exonuclease [11]. First, a hairpin probe with a phosphoric acid group at the end and methylene blue in the middle is fixed on the electrode surface. At this time, due to the rigid structure of the hairpin probe, the electroactive material is far from the electrode surface and the electrochemical signal is very low. The method provides a good idea for electrochemical amplification technology [12]. Lee et al. proved that the admittance of DNA-modified conductive polymer changed significantly after hybridization and proposed a DNA sensor based on measuring impedance. The electrochemical DNA biosensor based on hybridization indicator refers to the process of selecting appropriate electroactive substances to detect hybridization during the formation of double strands of DNA [13]. Xiao Y et al. [14] labeled one end of the DNA probe with derived methylene blue (MB) and characterized the hybridization process by detecting changes in the electrochemical signal of methylene blue before and after hybridization. The optical sensor designed with the principle of electroluminescence realizes the determination of polyromantic hydrocarbons in pure organic solvents and is an earlier report on the use of its for detection and analysis [15]. Electrochemiluminescence sensors generally require the introduction of luminescent labeling reagents [16]. However, with the continuous expansion of the sensor research, the types of electrochemiluminescence reagents are also increasing, and the structural design of the sensor has also been developed. Its application fields have been widely involved in DNA analysis, oncogene analysis, immune analysis, and environmental testing [17, 18].

With the continuous development of signal amplification technology and nanotechnology, more and more electrochemical sensors that combine nanotechnology and signal amplification technology are applied in the field of analysis [19, 20]. In this paper, combined with the Internet of Things technology, the construction of gold nanobiosensors and signal characteristic processing are carried out. The research purpose of this theory is to explore a simple, practical, and highly sensitive method for detecting melamine to establish a nonstandard, highly sensitive, and highly selective electrochemical method for DNA detection, which is useful for clinical testing, food safety, quarantine, and biological analysis. It has certain application prospects.

## 2. Gold Nanobiosensor

Metal nanoparticles have become one of the most attractive materials in biosensors due to their good optical, electrochemical, and catalytic properties. In recent years, the research on metal nanomaterials has also been continuously advancing [21]. Among them, signal amplification based on gold nanoparticles (AuNPs) and silver nanoparticles (AgNPs) is particularly effective in protein phosphorylation analysis [22]. Gold nanoparticles are also used as electrochemical detection signals to assist the construction of electrochemical sensors. Biotin-modified ATP is used as the source of phosphoric acid for protein kinase reaction. In the presence of protein kinase, the polypeptide substrate will be modified by biotin through the phosphorylation process [23]. At this time, the streptavidin-modified gold nanoparticles are added to the system. Due to the affinity between biotin and avidin, the gold nanoparticles are bound to the polypeptide substrate on the electrode surface. The electrochemical signal of oxidation of gold nanoparticles can be detected on the electrode surface by differential pulse voltammetry in electrochemical technology. In this paper, we studied the preparation of gold nanomaterials with large specific surface, strong conductivity, and biocompatibility and the construction of electrochemical sensors.

### 2.1. Preparation and Characterization of Gold Nanoparticles

With the continuous development of signal amplification technology and nanotechnology, more and more electrochemical sensors combining nanotechnology and signal amplification technology are applied in the field of analysis. Nanogold particles were prepared by reducing chloroauric acid by disodium citrate [24]. 100 mL of 0.01% HAuC14 solution was pipetted into a beaker, under vigorous stirring, after heating to boiling, 3 mL of newly prepared 1% disodium citrate solution was quickly added, and the solution was continued to boil and left until the color of the solution changed from dark blue to red. If it remains stable, a red nanogold particle solution can be obtained [25]. When the nanogold particle solution is cooled to room temperature, it is diluted to 100 mL, shaken well, characterized by using an ultraviolet-visible spectrophotometer, and stored in a refrigerator at 4°C.  Figure 1 shows a schematic diagram of the particle size distribution of AuNPs.

In the field of bioanalysis, in order to achieve the purpose of biomolecule detection, it is often necessary to modify the surface of gold nanoparticles. The most commonly used covalent modification of the surface of gold nanoparticles is basically divided into two methods [26].  Figure 2 depicts a schematic diagram of AuNP DLS.

The first is to form a self-assembled layer on the surface of gold nanometers through functional groups or derived functional groups of biomolecules. For example, in the gold nanoparticle solution prepared by the Ferns method, sodium citrate as a protective agent can form a stable protective film on the surface to control the growth of nanoparticles and inhibit the aggregation of nanoparticles. The gold nanoparticles were measured with an ultraviolet spectrophotometer to determine the peak position. Also, TEM (Transmission Electron Microscope) and DLS (Malvern Laser Particle Analyzer) were used to characterize the morphology and particle size distribution of the sample, and nanomeasure software was used to calculate and analyze the particle size results.

### 2.2. Melamine Detection

This section introduces the electrochemical signal detection of melamine based on DNA-modified gold nanoparticles. DNA1 was used as a capture probe to modify the surface of the gold electrode, and DNA2-AuNPs were used as a signal probe. Both of them contained T-rich sequences and did not hybridize themselves. The melamine and *T* can be combined through three hydrogen bonds [27, 28]. Therefore, in the presence of melamine, DNA1 can capture DNA2-AuNPs on the surface of the gold electrode. A nanogold particle is loaded with hundreds of DNA2 molecules, which can bind a large number of nail amine molecules through electrostatic adsorption, causing a significant increase in the chronoelectric signal, thereby realizing the detection of melamine.  Figure 3 shows the UV-Vis absorption spectra before and after modification of the reporter probe with gold nanoparticles.

Figure 3 shows the UV-visible spectra before and after the gold nanoparticles modified DNA2. The maximum absorption peak of the gold nanoparticles itself is 518 nm. When DNA2 is modified on the gold nanoparticles, its maximum absorption peak is red-shifted from 518 nm to 524 nm, indicating that DNA2 has been successfully modified into the gold nanoparticles.  Figure 4 depicts the UV-visible absorption spectra of the Le Reporter probe before and after surface modification of the gold nanoparticles.

It can be seen from Figure 5 that as the concentration of melamine increases from 0.4 NM to 400 NM, the chronoelectric signal gradually increases. It can be seen from the figure that as the concentration of melamine increases, *Q* gradually increases. It can be calculated that the lower detection limit of melamine is 0.5 NM, which is equivalent to 0.06 ng/ml. Figure 5 depicts the chronoelectric response results of different concentrations of melamine.

Therefore, the sensitivity of the sensor can meet the detection requirements. In addition, the sensitivity of the sensor is comparable or even higher than that of many methods reported so far. It has reduced cost. In addition, this ball can improve the current signal and enhance the sensitivity. Furthermore, the gold nanosensor significantly amplifies the electrochemical signal, so that the electrochemical aptameric sensor has higher sensitivity when used for melamine detection. Therefore, this strategy provides an option for the establishment of a cost-effective, media-free electrochemical biosensor and its use in amplifying the detection of other analyses.

## 3. Signal Feature Processing Based on the Internet of Things

By combining sensors with Internet of Things technology, melamine monitoring and signal characteristic processing can be carried out in real time. Signal amplification based on functionalized nanomaterials has attracted widespread attention in recent years. Functionalized nanomaterials can not only provide synergistic catalytic effects, electrical conductivity, and biocompatibility to accelerate signal transmission but also provide amplification recognition through the high load of the beacon to construct highly sensitive and specific sensors and are used in biological analysis. There are many applications in medical testing and other aspects [29]. Because of the unique biocompatibility and large specific surface area of nanomaterials, especially carbon materials and metal nanomaterials, it is very useful as a carrier to increase the amount of probes. Usually, nanomaterials are used as a base element to enrich target molecules or signal molecules to achieve signal amplification. Graphene oxide is used to immobilize a large number of electroactive substances, thiamin, to enhance the detection of DNA methylate activity. The linear range of response signal and methyl transferase activity is 0.1–450 U/mL, and the detection limit is as low as 0.05 U/ml. By constructing a conductive area between biomolecules and nanomaterials to provide a route for enhanced biological recognition, a conductive immunoassay sensor is constructed between two microelectrodes for protein determination, by forming a sandwich structure and depositing silver nanoparticles. The ions construct a conductive path between the two electrodes to achieve ultrasensitive detection of human immunoglobulin.

### 3.1. Detection Signal Amplification

For a specific weak photoelectric signal detection system, in the design process, the hardware platform of the detection system is required to have stable performance, high detection accuracy, and real-time performance to meet the requirements, so the matching and circuit matching must be considered when designing the detection system hardware. The major issue is the consistency of parameters in the circuit. This article designs the hardware circuit of the detection system for the weak photoelectric current signal. The hardware circuit composition block diagram is shown in Figure 6. The figure shows that the hardware composition of the weak photocurrent signal detection system in this article mainly includes front-end conditioning circuit, AD conversion circuit, and DSP control. There are four parts of the circuit and the communication interface circuit, of which the front-end conditioning part is mainly to amplify and filter the weak photocurrent signal. Figure 6 shows the hardware composition block diagram of the weak signal detection system.

The amplifier unit, that is, the amplifier in the amplification flowchart of this article, takes into account the pin requirements of dual input and dual output and adopts a fully differential structure, which has high gain, large unity gain bandwidth, large output swing, and high common mode rejection ratio as an advantage. The circuit structure adopted in this article is divided into bias circuit and main amplifier circuit. The amplifying circuit is divided into the first-stage amplification and the second-stage amplification. The first-stage mainly provides large gain, and the second stage not only provides amplification but also achieves large driving power and large swing. The weak photocurrent signal designed in this paper is designed based on the characteristics of the weak photoelectron current signal emitted by the ring sensor. The photoelectric conversion process needs to be designed in the weak photoelectric signal detection system. In addition, the influence of the experimental temperature on the entire detection process needs to be considered. The whole experiment process is further shielded to reduce the influence of ambient temperature on the test results.

### 3.2. Signal Feature Processing

In order to perform characteristic processing on the signal in the gold nanobiosensor, the Kalman filter algorithm is used in this paper. Before Kalman filtering is performed on the target system, an accurate mathematical model description of the target system is required, and the system that meets the conditions of this model can use the Kalman filter algorithm. A model that meets the following conditions is established and expressed with a linear stochastic difference equation:

(1) $$\begin{array}{c} x_{k}=Ax_{k-1}+Bu_{k-1}+w_{k-1},\\ z_{k}=Hx_{k}+v_{k}. \end{array}$$

*w*_*k*_ and *v*_*k*_ are white task positions that are not directly related, and both conform to an approximate normal distribution.

(2) $$\begin{array}{c} \left\{\begin{array}{c} p\left(w\right)⟶>\left(0,Q\right),\\ p\left(v\right)⟶>\left(0,Q\right). \end{array}\right. \end{array}$$

The calculation prototype of the Kalman filter algorithm is composed of the time update equation and the measurement update equation. There are two aspects. The a priori estimated value for the *k*-th step is ${\overset{\cdot }{x}}_{\overset{-}{k}}\in R^{n}$, which is estimated when the state before the *k*-th step is known. The posterior estimate of the *k*-th step is ${\overset{\cdot }{x}}_{k}\in R^{n}$, which is an estimate when the measured variables are known. Then, the errors of the prior and posterior estimates are

(3) $$\begin{array}{c} \bar{e_{k}}=x_{k}-{\overset{¯}{\dot{x}}}_{k},e_{k},\\ =x_{k}-{\dot{x}}_{k}, \end{array}$$

where A is the true state. Then, the covariance matrix of the prior estimation error and the covariance matrix of the posterior estimation error can be obtained as

(4) $$\begin{array}{c} \bar{P_{k}}=E\left[\bar{e_{k}}{\bar{e_{k}}}^{T}\right],\\ P_{k}=E\left[e_{k}e_{k}{}^{T}\right]. \end{array}$$

From this, the expression of the Kalman filter algorithm is obtained:

(5) $$\begin{array}{c} \bar{\dot{x}k}=\bar{\dot{x}k}+k\left(z_{k}-H\bar{\dot{x}k}\right). \end{array}$$

It can be seen that the value of the Kalman filter algorithm is a posterior estimated value, which is a weighted linear combination of the difference between the a priori estimated value ${\overset{\cdot }{x}}_{\bar{k}}$, the actual observation value *z*_*k*_, and the measured forecast $H{\overset{\cdot }{x}}_{\bar{k}}$. In the formula, $\left(z_{k}-H{\overset{\cdot }{x}}_{\bar{k}}\right)$ is the new observation value, also called the observation residual value. This value reflects the deviation between the actual observation value and the measured forecast value. If the observation residual value is 0, it means that the two are consistent. *K* is called the Kalman gain, which is

(6) $$\begin{array}{c} K_{k}=\bar{P_{k}}H^{T}{\left(H\bar{P_{k}}H^{T}+R\right)}^{-1},\\ =\frac{\bar{P_{k}}H^{T}}{H\bar{P_{k}}H^{T}+R}. \end{array}$$

The time update equation completes a priori estimation of the current state of the system and at the same time calculates the value of the current state variable and calculates the covariance value of the error. The state update equation uses the a priori estimation value of the system obtained by the time update equation to complete the posterior estimation after the current state is revised.

The time update equation is as follows.

The observation update equation is as follows:

(7) $$\begin{array}{c} K_{k}=P_{k}^{-}H^{T}{\left(HP_{k}^{-}H^{T}+R\right)}^{-1}. \end{array}$$

Because the nanosensor itself is a weak physiological electrical signal and it also receives interference from a variety of noises, noise reduction must be performed before *R*-wave recognition, and at the same time, useful information must be retained as much as possible. After noise reduction, we use Kalman filter to decompose the signal in 8 layers. According to the characteristics of the nanosensor and comparing the conditions of each layer after decomposition, the decomposition effect in the third layer is the best. Therefore, the sensitivity of the sensor can meet the detection requirements. In addition, the sensitivity of the sensor is comparable or even higher than that of many methods reported so far.

## 4. Conclusions

With the continuous development of signal amplification technology and nanotechnology, more and more electrochemical sensors combining nanotechnology and signal amplification technology are applied in the field of analysis. In this paper, we studied the preparation of gold nanomaterials with large specific surface, strong conductivity, and biocompatibility and the construction of electrochemical sensors. In this paper, a T-rich DNA probe is used as the identification element to develop a highly sensitive electrochemical biosensor for the detection of melamine. The sensor has good specificity and sensitivity, and the detection limit is as low as 0.5 NM. In addition, by combining sensors with the Internet of Things technology, melamine monitoring and signal characteristic processing can be carried out in real time. This model can easily achieve the purpose of accurate and quantitative analysis of melamine toxins and can be effective for food safety. In summary, the construction of a visual sensing system based on nanogold is an efficient and convenient sensing method, and it also provides new ideas for the detection and research of actual environmental biotechnology. In the future, we will combine other methods to analyze the current signal to effectively amplify the current signal and improve the sensitivity of the detection method, so that the sensor is expected to be used in clinical detection of other target proteins.

## Figures and Tables

**Figure 1:** Schematic diagram of AuNP particle size distribution.

**Figure 2:** Schematic diagram of AuNP particle DLS.

**Figure 3:** UV-Vis absorption spectra before and after modification of the reporter probe with gold nanoparticles.

**Figure 4:** UV-Vis absorption spectra of the reporter probe before and after surface modification of gold nanoparticles.

**Figure 5:** Timing electricity response results corresponding to different concentrations of melamine.

**Figure 6:** The hardware composition block diagram of the weak signal detection system.

## Data Availability

All data including supplementary materials are already in the manuscript.
